The article "Preparation of a pH‐responsive chitosan‐montmorillonite‐nitrogen‐doped carbon quantum dots nanocarrier for attenuating doxorubicin limitations in cancer therapy" was retracted in 2025. Reasons: duplicated images; duplicated data; unreliable results or conclusions; concerns about the data.

# Preparation of a pH‐responsive chitosan‐montmorillonite‐nitrogen‐doped carbon quantum dots nanocarrier for attenuating doxorubicin limitations in cancer therapy

**DOI:** 10.1002/elsc.202200016

**Published:** 2022-09-13

**Authors:** Erfan Rahmani, Mehrab Pourmadadi, Sohrab Ali Ghorbanian, Fatemeh Yazdian, Hamid Rashedi, Mona Navaee

**Affiliations:** ^1^ School of Chemical Engineering College of Engineering University of Tehran Tehran Iran; ^2^ Department of Life Science Engineering Faculty of New Science and Technologies University of Tehran Tehran Iran; ^3^ Department of Biotechnology School of Chemical Engineering College of Engineering University of Tehran Tehran Iran; ^4^ Pharmaceutical Sciences Research Center The Institute of Pharmaceutical Sciences (TIPS) Tehran University of Medical Sciences (TUMS) Tehran Iran; ^5^ Department of Pharmaceutical Biomaterials and Medical Biomaterials Research Center Faculty of Pharmacy Tehran University of Medical Sciences (TUMS) Tehran Iran

**Keywords:** carbon quantum dots, chitosan, doxorubicin, drug delivery, montmorillonite, pH‐responsive nanocarrier

## Abstract

Despite its widespread usage as a chemotherapy drug in cancer treatment, doxorubicin (DOX) has limitations such as short in vivo circulation time, low solubility, and poor permeability. In this regard, a pH‐responsive chitosan (CS)‐ montmorillonite (MMT)‐ nitrogen‐doped carbon quantum dots (NCQDs) nanocomposite was first developed, loaded with DOX, and then incorporated into a double emulsion to further develop the sustained release. The incorporated NCQDs into the CS‐MMT hydrogel exhibited enhanced loading and entrapment efficiencies. The presence of NCQDs nanoparticles in the CS‐MMT hydrogel also resulted in an extended pH‐responsive release of DOX over a period of 96 h compared to that of CS‐MMT‐DOX nanocarriers at pH 5.4. Based on the Korsmeyer‐Peppas model, there was a controlled DOX release at pH 5.4, while no diffusion was observed at pH 7.4, indicating fewer side effects. MTT assay showed that the cytotoxicity of DOX‐loaded CS‐MMT‐NCQDs hydrogel nanocomposite was significantly higher than those of free DOX (*p* < 0.001) and CS‐MMT‐NCQDs (*p* < 0.001) on MCF‐7 cells. Flow cytometry results demonstrated that a higher apoptosis induction achieved after incorporating NCQDs nanoparticles into CS‐MMT‐DOX nanocarrier. These findings suggest that the DOX‐loaded nanocomposite is a promising candidate for the targeted treatment of cancer cells.

**Abbreviations**
CS: chitosan
DLS: dynamic light scattering
DMEM: Dulbecco's Modified Eagle's Medium
DMSO: dimethylsulfoxide
DOX: doxorubicin
EDTA: Ethylenediaminetetraacetic acid
FBS: fatal bovine serum
FESEM: field emission scanning electron microscope
FTIR: Fourier transform infrared
GA: glutaraldehyde
LMW: low molecular weight
MMT: montmorillonite
MTT: 3‐(4, 5‐Dimethyl‐thiazol‐2‐yl)‐2, 5‐diphenyl‐tetrazolium bromide
NCQDs: nitrogen‐doped carbon quantum dots
PBS: phosphate buffer saline
PEG: polyethylene glycol
PVA: polyvinyl alcohol
XRD: X‐ray diffraction

The article "Preparation of a pH‐responsive chitosan‐montmorillonite‐nitrogen‐doped carbon quantum dots nanocarrier for attenuating doxorubicin limitations in cancer therapy" was retracted in 2025. Reasons: duplicated images; duplicated data; unreliable results or conclusions; concerns about the data.

## 1 INTRODUCTION

The incidence of cancer has dramatically increased over the last century, with 18.1 million new cases diagnosed in 2018 [1]. Several conventional methods, including chemotherapy, have been proposed to treat this deadly disease. Traditional chemotherapy is still being widely used in cancer treatment despite some drawbacks concerning specificity or selectivity [2]. Accordingly, various plant‐derived anticancer drugs with fewer side effects have received special attention [3]. The chemotherapy drugs derived from wild‐type strains of Streptomyces have been recently applied as an alternative cancer treatment [4].

Doxorubicin (DOX) belongs to an anthracycline class of drugs derived from *Streptomyces peucetius var. caesius* [5]. Based on its ability to promote reactive nitrogen species (RNS) and reactive oxygen species (ROS), DOX can be used for killing rapidly dividing cells albeit its toxicity toward normal cells [6]. DNA double‐strand breaks and the inhibition of DNA and RNA synthesis make DOX one of the most common natural (plant‐derived) drugs widely used in tumor therapy. DOX induces AMP‐activated protein kinase (AMPK) [7] and Bcl‐2/Bax [8] activation. It can also mitigate the problem of multidrug resistance of breast cancer cells by inhibiting the expression of P‐glycoprotein (Pgp) [9].

The above‐mentioned attributes of DOX make it suitable for cancer therapy, though it still has its limitations such as dose‐dependency, heart failure, poor solubility, and low bioavailability [10]. To surmount these constraints and cut down on dose administration, DOX entrapment into biodegradable polymeric carriers can be considered. Hydrogels have become popular among different drug delivery approaches for biodegradability, biocompatibility, non‐toxicity, and non‐immunogenicity [11]. However, hydrogel systems may encounter problems such as low entrapment of hydrophobic drugs in the hydrophilic hydrogel network and poor responses to stimuli. Hence, nanoparticles have been extensively incorporated into hydrogels to attain stimuli‐responsive hydrogel nanocomposites [12]. In other words, nanoparticles have transcended the limitations of hydrogels thanks to their ability to release encapsulated drugs in response to stimuli [13] as well as their potential to improve the entrapment efficiency of hydrophobic drugs in fabricated hydrogels [14].

The article "Preparation of a pH‐responsive chitosan‐montmorillonite‐nitrogen‐doped carbon quantum dots nanocarrier for attenuating doxorubicin limitations in cancer therapy" was retracted in 2025. Reasons: duplicated images; duplicated data; unreliable results or conclusions; concerns about the data.

In a recent study, hematite nanoparticles were added to chitosan‐polyvinylpyrrolidone hydrogels to delivery of doxorubicin to MCF‐7 cancer cells. Results have shown that adding hematite nanoparticles improves the loading and entrapment efficiencies of hydrogel nanocomposites. Besides, hematite‐based hydrogel nanocomposites were an excellent platform for anticancer application with reduced side effects and enhanced pH‐responsivity [15].

As mentioned by Liu [16], cancer cells are highly acidic compared to healthy cells. The acidic condition in the extracellular matrix of tumor cells is due to the abundance of lactic acid generated by the Warburg effect involved in the unrestrained proliferation of cancer cells through aerobic glycolysis [17]. Another recent study aimed to fabricate a pH‐responsive hydrogel nanocomposite to carry DOX to MCF‐7 cell lines. It has been confirmed that pH‐responsive delivery of chemotherapy drugs can effectively manage side effects and achieve the sustained release of therapeutics [18]. Nematollahi et al. developed chitosan‐polyvinylpyrrolidone‐γ‐alumina nanocomposite as a pH‐sensitive platform for the delivery of quercetin as the model drug. To develop this pH‐sensitive nanocomposite, nanoporous γ‐alumina was incorporated into chitosan‐polyvinylpyrrolidone hydrogel as the drug carrier. The results indicated that quercetin release was improved in acidic conditions (pH 5.4) compared to basic conditions (pH 7.4) [19].

Chitosan (poly‐[1, 2, 3, 4]‐β‐glucosamine, CS) is a polymeric hydrogel widely used in medicine and pharmacology [20] and the second natural polysaccharide together with cellulose deacetylated from chitin [21]. CS is a promising natural polymer for fabricating hydrogel‐based nanocarriers in a drug delivery system regarding its characteristics, that is, low toxicity, high biodegradability, biocompatibility, and pH‐responsivity [22]. Including primary amine and hydroxyl functional groups, CS can further establish hydrogen bonds with mucous membranes and epithelia. This provides CS‐based nanocarrier with effective bioadhesion and permeability. Furthermore, CS‐conjugated nanocarriers offer advantages like extended residence time and thus increased drug absorption [23]. These properties ensure the capability of CS as a good chemical in controlled drug delivery systems. Hydrogel structures, despite their many advantages, have a number of drawbacks in drug delivery, including inadequate homogeneity, paucity of multiresponsiveness, and unsatisfactory loading of hydrophobic medicines in hydrogels because of their hydrophilic nature. Eco‐friendly chemicals should thus be used as a reinforcing approach. The usage of naturally occurring nanoclay chemicals in the reinforcing method might be beneficial for enhancing polymer characteristics. When a polymer hydrogel is reinforced with proper nano‐clay additions, the discharge of a drug from a polymeric hydrogel may be regulated [24]. The physical, chemical, and mechanical characteristics of the polymeric hydrogel are affected when nano‐clay is added to this structure. While considering particular purposes, this modification of the physical and chemical properties of nano‐clay embedded polymeric hydrogels is critical. As a result, the inflating characteristics, heat withstandability, and mechanical durability of the augmented hydrogel may be tuned using nano‐clay embedded polymer hydrogel systems [25, 26].

The article "Preparation of a pH‐responsive chitosan‐montmorillonite‐nitrogen‐doped carbon quantum dots nanocarrier for attenuating doxorubicin limitations in cancer therapy" was retracted in 2025. Reasons: duplicated images; duplicated data; unreliable results or conclusions; concerns about the data.

Montmorillonite (MMT), a natural clay mineral, comprises two silica sheets covering one alumina sheet in between. The presence of oxide anions allows positively charged polymers such as CS to intercalate into the interlayer spaces of MMT, resulting in improved swelling and sustained release properties [27]. MMT has attracted substantial attention regarding its ability to improve the thermal stability and mechanical strength of nanocarriers [28]. These promising features have inspired the incorporation of MMT nanoclays into hydrogels for pH‐responsive drug delivery systems [29]. Despite the benefits of using nanoclays and hydrogels in drug delivery systems, low electrostatic repulsive forces between ionized groups and poor hydrophobic drug loading into hydrogels can compromise the efficacy of a pH‐responsive drug delivery platform. To tackle this serious challenge, carbon quantum dots (CQDs) nanoparticles of rich amino groups were incorporated into the fabricated hydrogel. Accordingly, the fabricated platform offered a pH‐responsive feature for CS‐MMT‐NCQDs interactions [30].

Notwithstanding the many advantages of employing hydrogels for drug delivery, drawbacks in hydrogel structures limit their widespread employment, including poor homogeneity, absence of multiresponsiveness, and insufficient hydrophobic medicines injection in hydrogels owing to their hydrophilicity. These faults may be remedied by adding nanomaterials to hydrogels, making hydrogels more useful in drug delivery [31]. Hydrogel nanocomposites are a favorable alternative for stimuli‐responsive directed drug delivery because of their smaller particle diameter, elevated surface region, controlled structure, and capacity to integrate hydrophobic compounds with magnetic, thermal, and electrical characteristics that can be recruited for sensitive discharge of entrapped medications [24].

**PRACTICAL APPLICATION**

- A novel method to synthesize a double emulsion‐based pH‐responsive system.
- The incorporation of NCQDs was significantly effective in the increase of drug loading and entrapment efficiency.
- The fabricated CS‐MMT‐NCQDs hydrogel nanocomposite exhibited targeted and controlled release of DOX.
- The nanocarrier exhibited higher apoptosis induction after the incorporation of NCQDs nanoparticles into CS‐MMT‐DOX.

The article "Preparation of a pH‐responsive chitosan‐montmorillonite‐nitrogen‐doped carbon quantum dots nanocarrier for attenuating doxorubicin limitations in cancer therapy" was retracted in 2025. Reasons: duplicated images; duplicated data; unreliable results or conclusions; concerns about the data.

NCQDs, also known as semiconducting nanoparticles, are small carbon nanoparticles (less than 10 nm in size) with unique optical properties such as photostability, non‐photobleaching, signal brightness, and resistance to simultaneous multi‐color fluorescence excitation [32]. On the other hand, their optical and electronic properties can be tuned to emit a broad range of visible regions [33]. Extensive studies have been conducted on semiconducting quantum dots, with recent attention and advances in nanoparticle surface chemistry to seize new opportunities for developing pH‐responsive nanocarriers using biopolymers and NCQDs [34]. Zavareh et al. fabricated chitosan‐carbon quantum dots‐aptamer as a carrier of 5‐fluorouracil. Based on their results, the fabricated nanocarrier retained the release of 5‐fluorouracil in the normal physiological condition (pH 7.4), while releasing almost the entire drug in the tumor microenvironment (pH 5.4) [35]. The nanomaterials of CQDs were examined by Cutrim and his colleagues during the discharge of 5‐FU [36]. Antitumor 5‐FU was self‐assembled onto carbon quantum dots in this work to provide a unique medication delivery method. 5‐FU‐CQD nanoconjugate may improve tumor treatment by lowering the cytotoxicity towards healthy tissues associated with free 5‐FU, according to this research outcome. This allows for the minimization of unpleasant symptoms while retaining the clinical efficacy of 5‐FU. Regarding the delivery of DOX covalently linked with carbon dots (CDs) functionalized by nuclear localization signal peptide (NLS‐CDs) via a pH‐responsive hydrazone connection, Yang et al. [37] developed an innovative nucleus‐targeted nanocomplex. More late apoptotic cells were seen in cells exposed to DOX‐CQDs than those treated with unbound DOX. This might be a result of the manufactured complexes' enhanced sustained‐release characteristics. Furthermore, the consolidation of nanocomplex framework is maintained via pH‐responsive hydrazone connections, resulting in a lower accumulated discharge of CQDs‐DOX at pH 7.4 than pH 5.4.

A water‐in‐oil‐in‐water (W/O/W) double nanoemulsion was prepared following the procedure reported in the previous work [38]. Incorporating the fabricated nanocomposite into the W/O/W double nanoemulsion is an advance on hydrogel nanocomposites in terms of prolonging the drug release time. Indeed, the thin layer of the oil phase between internal and external aqueous phases functions as a barrier to hydrophobic DOX release from the internal aqueous phase [39]. To form a primary emulsion (W/O), a drug‐loaded hydrogel nanocomposite was added to a lipophilic emulsifier, playing the role of emulsion stabilizer. The primary emulsion (W/O) was dispersed in a second aqueous phase by applying a hydrophilic emulsifier to stabilize an oil‐water interface. The resultant solution was then stirred to form a W/O/W double nanoemulsion encapsulated DOX‐loaded hydrogel nanocomposite.

The article "Preparation of a pH‐responsive chitosan‐montmorillonite‐nitrogen‐doped carbon quantum dots nanocarrier for attenuating doxorubicin limitations in cancer therapy" was retracted in 2025. Reasons: duplicated images; duplicated data; unreliable results or conclusions; concerns about the data.

In this study, DOX was loaded into a pH‐responsive CS‐MMT‐NCQDs nanocomposite and then encapsulated in a fabricated nanocarrier by the W/O/W emulsification method. Moreover, our research aimed to study the antitumor effects of the fabricated pH‐responsive nanocarrier on MCF‐7 breast cancer cells. All in all, the main objectives of this study were to control drug release, enhance drug loading, and achieve apoptosis induction. To the best of our knowledge, this is an original strategy that benefits from the mentioned materials to fill the existing gaps in DOX cancer therapy. Simultaneously, our study yields satisfactory results regarding improved drug loading, strong cytotoxicity, and sustained release of DOX.

## 2 MATERIALS AND METHODS

### 2.1 Materials

LMW chitosan (CS, 50–190 kDa, degree of deacetylation 75%–85%), acetic acid, sodium montmorillonite (MMT, cation exchange capacity 92 meq/100 g of clay), diammonium hydrogen citrate (C_6_H_14_N_2_O_7_), polyvinyl alcohol (PVA), absolute ethanol, and glutaraldehyde (GA) were obtained from Merck. Doxorubicin (DOX) was purchased from Sigma–Aldrich. The other chemicals with analytical grade were used without further purification. Distilled water was purified with a Milli‐Q water purification system (18.2 MΩ cm, PureFlow Inc.) and utilized for all solutions.

### 2.2 NCQDs synthesis

NCQDs were prepared through a hydrothermal method according to the previously reported literature [40]. Firstly, 2 g of diammonium hydrogen citrate was dispersed in 75 mL deionized water. Then, the solution was carried into a Teflon‐lined autoclave with 100 mL capacity. The sealed tank was heated and maintained at 120˚C for 10 h in an oven. After finishing the reaction, the autoclave was naturally cooled down. Finally, the mixture was centrifuged at 10,000 rpm for 10 min to collect NCQDs. The concentration of synthesized NCQDs from the citrate source was calculated to be at about 26.66 mg mL^−1^.

### 2.3 Synthesis of CS‐MMT‐NCQDs hydrogel

CS‐MMT hydrogel was prepared applying the emulsion method by Samadi et al. [41]. In the first stage, 2% (w/v) CS nanoparticles were slowly added into 3 mL of aqueous acetic acid 2% (v/v)10000 making use of a magnetic stirrer (60˚C, 500 rpm) to reach a homogeneous solution. The 2% (v/v) acetic acid solution was added into the CS solution at 40°C and homogenized with a magnetic stirrer (∼500 rpm) for about 1 h. In the next stage, MMT was initially dissolved in deionized water to reach 1% (w/v) before adding to the prepared mixture. The addition of MMT to the prepared homogeneous solution under stirring conditions (∼500 rpm) resulted in non‐covalent bonds between CS and MMT. The prepared NCQDs were quickly injected into the CS‐MMT hydrogel at room temperature and stirred (∼500 rpm) for 15 min. In the final stage, the hydrogel was sonicated for about 10 min using a probe sonication and ultrasound to get a homogenous solution with the uniform dispersion of NCQDs nanoparticles.

The article "Preparation of a pH‐responsive chitosan‐montmorillonite‐nitrogen‐doped carbon quantum dots nanocarrier for attenuating doxorubicin limitations in cancer therapy" was retracted in 2025. Reasons: duplicated images; duplicated data; unreliable results or conclusions; concerns about the data.

### 2.4 Incorporation of DOX in CS‐MMT‐NCQDs hydrogel

For the loading of DOX in the CS‐MMT‐NCQDs hydrogel films, 70 µL DOX (2 mg mL^−1^) was first dissolved in absolute ethanol and then added drop‐wise into the hydrogel (30 mL) under vigorous stirring conditions (∼600 rpm). The drug‐loaded nanoparticles were obtained using GA as a cross‐linker. In this step, after the addition of 0.02% (v/v) GA into the solution, the mixture was stirred (∼125 rpm) for about 1 h to reach a homogenous CS‐MMT‐NCQDs hydrogel solution for DOX incorporation. The structure of fabricated hydrogel nanocomposite is shown in Figure 1. In next step, DOX loaded nanocarriers (10 mL) were drop‐by‐drop loaded and emulsified into 30 mL of liquid paraffin containing 2% (w/v) span 80 emulsifier in a hydrophobic phase. The resultant solution was stirred (∼250 rpm) to form a primary emulsion (W/O). Here, the fabricated nanoemulsion was separated from hydrophobic phase using hydrophilic phase containing 30 mL PVA 1% (v/v). The lower density of the hydrophobic phase made it floated above the hydrophilic phase and removable by the use of a laboratory sampler. The addition of this particular hydrophilic phase caused the fabricated nanoemulsion sedimentation in the remaining hydrophilic phase. The sedimentation of the fabricated nanoemulsions was based on the high affinity of their external aqueous phase toward the hydrophilic phase. The remaining hydrophilic phase was then centrifuged at 3500 rpm for 10 min. In the last step, the nanocarriers were left in liquid nitrogen for 5 min before transferring into the freeze dryer.

**FIGURE 1:** Schematic representation of cross‐linked CS‐MMT‐NCQDs‐DOX hydrogel nanocomposite

### 2.5 Characterization

X‐ray diffraction (XRD) pattern was obtained from the samples by X‐ray diffraction (XRD, PHILIPS, PW1730, Netherlands) using Cu/K*α* (1.54056 Å,40 kv,30 Ma) in the 2θ range from 5˚ to 80˚ (0.05 deg step size and 1 s per step). The data were collected using HighScore Plus version3. To determine interactions between components in the samples of CS‐MMT, CS‐MMT‐NCQDs, CS‐MMT‐NCQDs‐DOX, Fourier transform infrared (FTIR) spectrophotometry were recorded from the samples on a Thermo AVATAR FT‐IR spectrometer (Chicago, Illinois, US) at room temperature. The scanning range of the spectrum was between 600 and 4000 cm^−1^. Employing MALVERN ZEN3600 (Malvern, UK), dynamic light scattering (DLS) and zeta potential measurements were respectively done for determining the average size distribution and the surface charge of nanoemulsions. Field‐emission scanning electron microscopy (FESEM, TESCAN MIRA III, Brno, Czechia) was also used to characterize the CS‐MMT‐NCQDs‐DOX morphology. The sonication of solutions was carried out before conducting experiments.

The article "Preparation of a pH‐responsive chitosan‐montmorillonite‐nitrogen‐doped carbon quantum dots nanocarrier for attenuating doxorubicin limitations in cancer therapy" was retracted in 2025. Reasons: duplicated images; duplicated data; unreliable results or conclusions; concerns about the data.

### 2.6 Doxorubicin entrapment and loading efficiency measurement

To ascertain efficiency of DOX entrapment and loading, 1 mg of CS‐MMT‐NCQDs‐DOX nanocomposite was added to 1 mL phosphate buffer saline (PBS), then the prepared solution was supplemented with 1 mL of ethyl acetate. In order to extract ethyl acetate, the mixture was shaken. UV‐Vis spectrophotometer quantified the content of free DOX in the ethyl acetate phase at 485 nm [42]. The efficiency percentages of DOX entrapment and loading were calculated using Equations (1) and (2) [15].

(1) $$\begin{array}{ccc} & & \mathrm{Entrapment}\;\mathrm{efficiency}\left(\%\right)=\\ & & \;\frac{\left(\mathrm{Total}\;\mathrm{amount}\;\mathrm{of}\;\mathrm{DOX}\right)-\left(\mathrm{Free}\;\mathrm{amount}\;\mathrm{of}\mathrm{DOX}\right)}{\left(\mathrm{Total}\;\mathrm{amount}\;\mathrm{of}\;\mathrm{DOX}\right)} \end{array}$$

(2) $$\begin{array}{ccc} & & \mathrm{Loading}\;\mathrm{efficiency}\left(\%\right)=\\ & & \;\frac{\left(\mathrm{Total}\;\mathrm{amount}\;\mathrm{of}\;\mathrm{DOX}\right)-\left(\mathrm{Free}\;\mathrm{amount}\;\mathrm{of}\;\mathrm{DOX}\right)}{\left(\mathrm{Total}\;\mathrm{amount}\;\mathrm{of}\;\mathrm{Nanocomposite}\right)} \end{array}$$

### 2.7 In vitro drug release study

The release of DOX from CS‐MMT‐NCQDs nanocarrier was studied utilizing the dialysis bag diffusion method for two different media of phosphate buffer media at two different pH levels of 5.4 and 7.4 in a water bath set to 37˚C. The content of 1 mL of CS‐MMT‐NCQDs‐DOX nanocarrier was added into a dialysis bag which was immersed in 15 mL of phosphate buffer medium containing 20% (v/v) ethanol at pH 5.4 and pH 7.4 at 37˚C. 20% (v/v) ethanol was used as a solvent to dissolve the poorly soluble drug, DOX. At adopted time intervals, 300 µL of samples were extracted and substituted with an equal amount of fresh PBS buffer to retain a constant volume. The released DOX content in the buffer was measured by a spectrophotometer at 485 nm [42]. The quantity of released DOX was calculated employing the equation below:

(3) $$\mathrm{DOX}\;\mathrm{released}\left(\%\right)=\frac{\left[\mathrm{DOX}\right]\mathrm{rel}}{\left[\mathrm{DOX}\right]\mathrm{load}}*100$$

Where [DOX]load refers to the quantity of doxorubicin encapsulated in the nanocarrier, and [DOX]rel represents the quantity of doxorubicin released from the nanocarrier.

The article "Preparation of a pH‐responsive chitosan‐montmorillonite‐nitrogen‐doped carbon quantum dots nanocarrier for attenuating doxorubicin limitations in cancer therapy" was retracted in 2025. Reasons: duplicated images; duplicated data; unreliable results or conclusions; concerns about the data.

### 2.8 Release kinetics

To assess the mechanism of drug release at pH 7.4 and pH 5.4, the release data of DOX was fitted to empirical and semi‐empirical models, including first‐order (Equation 4), Higuchi (Equation 5), Hixson‐Crowell (Equation 6), Baker (Equation 7), and Korsmeyer‐Peppas (Equation 8). Where *M_t_* is the cumulative release of the drug at time *t*, *M_∞_* is the cumulative release of the drug at the equilibrium state; *f_t_* is the portion of drug released at time *t*, *f _t_*_,max_ is the greatest portion of drug released during a process; and *K*_1_, *K_p_*, *K_β_*, *K_C_*, and *K_H_* are the rate constants of the Equations (4), (5), (6), (7), and (8), respectively. We fitted the data to the models to determine *R* ^2^ for each model. The best fitting regression model entails mere consideration of meaningful parameters. The equations of the mentioned models used for determining the release mechanism are listed below.

(4) $$f_{t}=\;f_{t,\max}*\left(1-\exp\left(-K_{1}*t\right)\right)$$

(5) $$\left(\frac{M_{t}}{M_{\infty }}\right)=K_{P}\;*\sqrt{t}$$

(6) $$\sqrt[{3}]{1-f_{t}}=\;1-K_{\beta }*t$$

(7)

(8) $$\frac{M_{t}}{M_{\infty }}=K_{H}\;*t^{n}$$

### 2.9 Cytotoxic analysis of the fabricated nanocarrier

The 3‐(4,5‐dimethylthiazol‐2‐yl)‐2,5‐diphenyltetrazolium bromide (MTT) assay was employed to study the cytotoxicity of CS‐MMT‐NCQDs, CS‐MMT‐NCQDs‐DOX, and free DOX on MCF‐7 breast cancer cell line. The concentration of free DOX was 4.8 µg mL^−1^, which is equal to DOX concentration in the fabricated CS‐MMT‐NCQDs‐DOX and CS‐MMT‐DOX nanocarriers according to the loading efficiency of DOX in the nanocarrier. MCF‐7 cells were cultured in 200 µL of Dulbecco's Modified Eagle's Medium (DMEM) media added to a 96‐well tissue culture plate at a density of 5 × 10^3^ per well. The cells were incubated for 24 h to which the samples were added and incubated for 48 h when 80% of the surface of culture vessel was coated. The cells were cultured as control without any treatment in DMEM basic medium including 10% fatal bovine serum (FBS) and 1% penicillin/streptomycin for 24 h. After 72 h, 50 µL of 5 mg mL^−1^ MTT was added to each well with the plates incubated for 4 h at 37˚C. To dissolve the purple formazan crystals, the media were elicited and substituted with 200 µL of dimethylsulfoxide (DMSO). The plates were stirred for about 10 min, and optical density was read at 570 nm by a microplate reader. Cell viability percentage was measured applying Equation (9):

(9) $$\begin{array}{c} \begin{array}{ccc} & & \;\mathrm{Cell}\;\mathrm{viability}\left(\%\right)=\\ & & \frac{\mathrm{Absorbance}\;\mathrm{of}\;\mathrm{well}\;\mathrm{with}\;\mathrm{nanoparticles}\;\mathrm{at}\;570\;\mathrm{nm}}{\mathrm{Absorbance}\;\mathrm{of}\;\mathrm{well}\;\mathrm{without}\;\mathrm{nanoparticles}\;\mathrm{at}\;570\mathrm{nm}}*100 \end{array} \end{array}$$

The article "Preparation of a pH‐responsive chitosan‐montmorillonite‐nitrogen‐doped carbon quantum dots nanocarrier for attenuating doxorubicin limitations in cancer therapy" was retracted in 2025. Reasons: duplicated images; duplicated data; unreliable results or conclusions; concerns about the data.

### 2.10 Cell apoptosis analysis

First, MCF‐7 cells were plated in a 6‐well plate at a density of 3 × 10^5^. The plates were then incubated for 24 h. Here, the cells were treated with CS‐MMT, CS‐MMT‐NCQDs, CS‐MMT‐DOX, CS‐MMT‐NCQDs‐DOX, and free DOX. There was an equivalent concentration of drug 4.8 µg mL^−1^ in nanocarriers. Next, the cells were left for incubation for the next 72 h. Those untreated cells were taken as control group. After being harvested by trypsin/Ethylenediaminetetraacetic acid (EDTA) 25%, the cells were washed with PBS and suspended in 100 µL binding buffer. The cells were stained with Propidium iodide (PI) and Annexin V‐fluorescein and kept in the dark for 15 min. Eventually, a flow cytometer was employed to examine the samples.

## 3 RESULTS AND DISCUSSION

### 3.1 Characterization

#### 3.1.1 FTIR spectroscopy

FTIR analysis was conducted in order to identify chemical bonds between CS, MMT, NCQDs, and DOX. FTIR spectra for CS, CS‐MMT, CS‐MMT‐NCQDs, and CS‐MMT‐NCQDs‐DOX are represented in Figure 2. In the FTIR spectrum of CS, the band at 1020 cm^−1^ is ascribed to the bending vibrations of amide I groups. The band at 1150 cm^−1^ corresponds to C–O stretching present in CS [43]. N–H binding of amide II was accredited to the band at 1580 cm^−1^ [44]. The absorption band at around 1370 cm^−1^ can be ascribed to the symmetrical angular deformation of CH_3_ [45]. Carbonyl stretching vibration of the secondary amide and C–H stretching were verified by the existence of bands at 1680 and 2850 cm^−1^, respectively, as described in previous studies [19, 43]. A wide band in the region 3000–3560 cm^−1^ is related to N–H and O–H stretching [43].

**FIGURE 2:** The FTIR spectra of CS, CS‐MMT, CS‐MMT‐NCQDs, and CS‐MMT‐NCQDs‐DOX

The FTIR spectra of NCQDs showed unique bands in the 1045 cm^−1^ (N–C), 1600 cm^−1^ (C = O), and 2920 cm^−1^ (C–H) ranges [30]. Because of this, it can be assumed that the NCQD‐related band resulting from comparable research by Liu and colleagues [46] may be attributed to the citrate source. NCQDs were shown to be hydrophilic and stable in another work by Yao Lu et al., and this was linked to the vibration of OH/NH_2_ in the wide absorption regions at 3368–3564 cm^−1^. The C = O vibration was shown to be responsible for absorbance at 1547 cm^−1^ and 1706 cm^−1^ [47].

The article "Preparation of a pH‐responsive chitosan‐montmorillonite‐nitrogen‐doped carbon quantum dots nanocarrier for attenuating doxorubicin limitations in cancer therapy" was retracted in 2025. Reasons: duplicated images; duplicated data; unreliable results or conclusions; concerns about the data.

In the FTIR spectra of CS‐MMT, CS‐MMT‐NCQDs, and CS‐MMT‐NCQDs‐DOX, all distinguishing bands of CS were observed. The wide band at 1580 cm^−1^ in CS, corresponding to the NH bending (amide II), was shifted toward lower frequency (1541 cm^−1^ in CS‐MMT, 1534 in CS‐MMT‐NCQDs, and 1520 in CS‐MMT‐NCQDs‐DOX) [48]. In the FTIR spectrum of CS‐MMT, the band at 1541 cm^−1^ became broader, indicating an electrostatic interaction between OH^−^ groups of MMT and N–H groups of CS. In the FTIR spectrum of CS‐MMT, the intensity of the band at 2850 cm^−1^ ascribed to C–H stretching vibration increased, indicating the crosslinked structure of the CS‐MMT nanocarrier. The FTIR of CS‐MMT‐NCQDs and CS‐MMT‐NCQDs‐DOX showed all functional bands of NCQDs nanoparticle. The decrease in the intensity of some of the NCQDs bands (1400 to 1373, 1600 to 1534, 2920 to 2856, and 3420 to 3348) can be ascribed to the interaction between CS‐MMT and NCQDs. In the FTIR spectrum of CS‐MMT‐NCQDs‐DOX, the band at 3284 cm^−1^ attributed to N–H and O–H stretching showed decreased intensity. This could be due to electrostatic interactions among the protonated amine groups of DOX and components in the fabricated nanocomposite, verifying the successful loading of DOX into CS‐MMT‐NCQDs nanocarrier [49]. Additionally, strong interaction with the drug resulted in a higher dissolution rate [50].

#### 3.1.2 XRD analysis

XRD was performed to further confirm the nanocarrier formation. The XRD patterns of CS, CS‐MMT, CS‐MMT‐NCQDs, and CS‐MMT‐NCQDs‐DOX are presented in Figure 3. The diffraction band of CS appeared at 2θ of 20.14°. The band at 2θ = 20.14° is related to the hydrated crystal of CS. This obtained value is in line with that reported in the previous literature [51]. After the addition of MMT to CS, the diffraction was found at 14.40° (2θ). In agreement with previous studies [48, 52], the initial band intensity in CS was much broader compared to that of CS‐MMT, suggesting the amorphous nature of silica sheets in MMT. The band shift from a higher diffraction angle (20.14°) to a lower diffraction angle (14.40°) decreased the band intensity of CS‐MMT compared to CS. This strongly suggests the intercalation of CS into MMT interlayer spacing [53]. In the XRD pattern of NCQDs, an amorphous carbon‐based chemical may be identified by a single wide diffraction band at 24.1° [54]. Figure 3 shows the XRD patterns of CS‐MMT‐NCQDs and CS‐MMT‐NCQDs‐DOX. There is a drop in the strength of the specific NCQDs band at 2θ = 24.1°. The integration of NCQDs nanostructures into the CS‐MMT and CS‐MMT‐DOX matrixes was confirmed by this finding. The XRD of the drug‐loaded nanocarrier showed a new band at a lower angle of 11.30° compared to the XRD of CS‐MMT‐NCQDs that showed a band at 2θ = 12.45°, showing the successful load of the drug in the nanocarrier. Moreover, the XRD pattern of CS‐MMT‐NCQDs‐DOX displayed no characteristic band for DOX from which it can be further inferred that the drug was successfully loaded into the nanocarrier [55]. The present results provide confidence for the FTIR analysis.

The article "Preparation of a pH‐responsive chitosan‐montmorillonite‐nitrogen‐doped carbon quantum dots nanocarrier for attenuating doxorubicin limitations in cancer therapy" was retracted in 2025. Reasons: duplicated images; duplicated data; unreliable results or conclusions; concerns about the data.

**FIGURE 3:** The XRD patterns of CS, CS‐MMT, CS‐MMT‐NCQDs, and CS‐MMT‐NCQDs‐DOX

#### 3.1.3 FESEM, zeta potential, and DLS studies of drug‐loaded nanocarriers

The morphological analysis of the nanocarriers loaded with DOX is demonstrated in Figure 4. Nanocarriers have a well‐defined spherical shape. The dark entities on the surface of fabricated nanocarriers representing the intersection of MMT layers were clearly visible at a 5 µm scale in Figure 4 [56]. Further, the surface homogeneity of the nanocarrier can be ascribed to the compatibility between the nanocarrier components. Uniformity in both size and shape is visible at a 20 µm scale, corroborating monodisperse nanocarriers in nanoscale. There is a satisfactory agreement between our FESEM images and reported morphology of CS‐MMT microspheres for fertilizer delivery systems by dos Santos et al. [57]. Zavareh et al. introduced CS‐CQDs‐aptamer nanocarrier for pH‐responsive drug delivery [35]. In the present work, the polydispersity, smooth, and spherical shape of the fabricated nanocarriers reinforced our morphological analysis.

**FIGURE 4:** FESEM image of CS‐MMT‐NCQDs nanocarrier loaded with DOX

The size distribution profile and poly disparity of CS‐MMT‐NCQDs‐DOX nanocarriers were determined using DLS analysis. The DLS results showed a peak intensity of nearly 100% with an X‐average value of 276.80 nm and also monodisperse distribution. Monodispersity herein refers to the uniform nanocarriers in both size and shape, which is consistent with the FESEM images. As evidenced by Mazzotta [58], the distribution inside capillaries and the accumulation in the tumor site are efficient for nanocarriers following the EPR (enhanced permeability and retention) effect.

The article "Preparation of a pH‐responsive chitosan‐montmorillonite‐nitrogen‐doped carbon quantum dots nanocarrier for attenuating doxorubicin limitations in cancer therapy" was retracted in 2025. Reasons: duplicated images; duplicated data; unreliable results or conclusions; concerns about the data.

In order to test the stability of nanocarriers, zeta potential measurement was performed. Particles with a zeta potential of more than +30 mV are considered stable. Zeta potential was estimated at +31.5 mV, confirming the stability of nanocarriers. This is consistent with the fact that no aggregation was found after the nanocarriers were left standing for 1 month. Besides, positive zeta potential can improve the uptake of cancerous cells as indicated by Dou [59].

### 3.2 DOX loading and entrapment efficiency

Among other factors, a fabricated nanocarrier efficacy is highly dependent on loading as well as entrapment efficiency because the effectiveness of a drug delivery system compromises with poor loading capacity [60]. Furthermore, as mentioned earlier, DOX direct admission is restricted by poor solubility and limited bioavailability. As a result, improving DOX loading as well as entrapment efficiency takes a giant leap in drug administration methods. Equations (1) and (2) have been used to calculate drug entrapment and loading efficiencies after determining its free or unentrapped quantity in the ethyl acetate phase. The loading efficiency was determined as 37% in CS‐MMT‐NCQDs and 49% in CS‐MMT‐NCQDs‐DOX, indicating drug loading improvement by adding NCQDs into the nanocarrier (Table 1). This improvement was dependent on the interactions between the –NH_2_ groups of NCQDs and Si–OH groups of MMT, –OH groups of NCQDs and amine groups of CS, and the –OH and –NH_2_ groups of NCQDs and DOX, originating from the addition of NCQDs into the CS‐MMT‐DOX nanocarrier. Interestingly, if we now turn to FTIR results, a decrease is observed in the intensity of a band related to N–H and O–H stretching after the drug loading in the nanocarrier. It can be proposed that the interaction between NCQDs and DOX is partly responsible for FTIR lower band intensity and thus greater loading efficiency. This finding fairly well correlates with that of Peng [61]. The result represents a clear improvement in current studies regarding drug loading in pH‐responsive nanocarriers.

**TABLE 1:** Influence of NCQDs on DOX loading and entrapment efficiencies

	**CS‐MMT**	**CS‐MMT‐NCQDs**	**Change (%)**
Loading (%)	37	49	+12
Entrapment (%)	68	91	+31

Li et al. prepared pH‐responsive pullulan‐DOX conjugate nanoparticles for hepatic targeting with a maximum drug loading efficiency of 28.5% [62]. Luan et al. synthesized hyaluronic acid‐based pH‐responsive nanogels for the delivery of DOX to tumor cells. The nanocarriers with a loading efficiency of 12.5% could induce cell apoptosis [63]. Xie et al. used the hybrid cluster bombs of PEGylated chitosan for targeted tumor‐specific DOX delivery and MR imaging. The nanocarriers showed a drug loading percentage of 24.3% [64].

The article "Preparation of a pH‐responsive chitosan‐montmorillonite‐nitrogen‐doped carbon quantum dots nanocarrier for attenuating doxorubicin limitations in cancer therapy" was retracted in 2025. Reasons: duplicated images; duplicated data; unreliable results or conclusions; concerns about the data.

The entrapment efficiency of DOX was 68% in CS‐MMT nanocarrier and improved to 91% in CS‐MMT‐NCQDs (Table 1). Based on redox degradable polymer, Xiong et al. prepared pH‐responsive micelles to load DOX in the hydrophobic core and gold nanoparticles in the hydrophilic shell for computed tomography imaging and controlled drug release with an entrapment efficiency of 48.4% [65]. The entrapment efficiency of DOX in the CS‐MMT‐NCQDs nanocarrier is close to that reported for pH‐responsive mesoporous silica nanoparticles coated with polydopamine (PDA) and polyethylene glycol (PEG) in breast cancer therapy [ 66 ]. Emami Gerami et al. studied the effect of hematite (α‐Fe2O3) nanoparticles on chitosan (CS)/polyvinylpyrrolidone (PVP) for doxorubicin delivery. It was stated that the addition of hematite (α‐Fe2O3) nanoparticles resulted in higher drug loading and entrapment efficiency percentages. It was concluded that the use of hematite (α‐Fe2O3) nanoparticles increased drug encapsulation and drug loading respectively from 73% to 89% and 46% to 52% [15]. The loading and entrapment efficiency are compared with previous studies in Table 2.

**TABLE 2:** A summary of results presented in previous works and the present work

Drug delivery platforms for doxorubicin delivery	Loading%	Entrapment%	Reference
Pullulan‐DOX conjugate nanoparticles	28.5	–	[55]
Hyaluronic acid‐based pH‐responsive nanogels	12.5	–	[56]
Hybrid cluster bombs of PEGylated chitosan	24.3	–	[57]
Micelles based on redox degradable polymer	–	48.4	[58]
Mesoporous silica nanoparticles coated with polydopamine (PDA) and polyethylene glycol (PEG)	–	95.63	[59]
Chitosan (CS)/polyvinylpyrrolidone (PVP)/hematite (α‐Fe_2_O_3_) nanocomposites	52	89	[15]
Chitosan (CS)/polyvinylpyrrolidone (PVP) nanocomposites	46	73	[15]
DOX‐loaded CS‐MMT‐NCQDs nanocomposite	49	91	This work

### 3.3 Release of DOX

We opted for the dialysis method to investigate pH‐triggered and sustained release of DOX from CS‐MMT‐NCQDs and CS‐MMT nanocarriers at pH 5.4 and pH 7.4 at 37˚C over 96 h (Figure 5). We chose pH 5.4 and pH 7.4 in order to simulate tumor microenvironment and normal tissue, respectively. In previous studies, the pH responsivity of NCQDs and CS were investigated [67, 68]. In the present study, the rational approach is to see the pH‐controlled release of DOX from CS‐MMT and CS‐MMT‐NCQDs nanocarriers. As Figure 5 depicts, the release profiles were characterized by an initial burst in the first 12 h followed by a sustaining release. The initial burst release might be ascribed to the quick release of drug adsorbed on the surface of nanocarriers. Additionally, the rapid swelling of the nanocarriers and the high concentration gradient of the drug could be due to the fast diffusion of the drug in the first 12 h [69].

The article "Preparation of a pH‐responsive chitosan‐montmorillonite‐nitrogen‐doped carbon quantum dots nanocarrier for attenuating doxorubicin limitations in cancer therapy" was retracted in 2025. Reasons: duplicated images; duplicated data; unreliable results or conclusions; concerns about the data.

**FIGURE 5:** In vitro release profile of DOX loaded CS‐MMT‐NCQDs nanocarrier and CS‐MMT without NCQDs in pH 5.4 and pH 7.4 at 37˚C at predetermined time intervals using the dialysis method

Under acidic circumstances, the accumulated discharge proportion was consistently much higher than the typical level. CS‐MMT‐DOX discharges doxorubicin at a rate of 74% and 64% at pH values range from 5.4 to 7.4, respectively, after 48 h of incubation. Higher medication is released from the CS‐MMT‐DOX nanocomposite under acidic settings (pH 5.4) in contrast to basic conditions (pH 7.4), which is due to poorer H‐bonding and electrostatic interaction between CS and MMT nanocomposites. At pH 5.4, the amino groups on the DOX and CS are protonated, accelerating the disintegration of polymeric hydrogel chains. This shows that the CS‐MMT nanocarrier is pH‐responsive in nature. In agreement with the findings of Depan et al. [70], this might be the result of interconnections between MMT layers.

The release of the drug from CS‐MMT nanocarrier was 47% within 24 h at pH 5.4, whereas 66% of the drug was released from CS‐MMT‐NCQDs within 24 h at pH 5.4. As shown in Figure 5, the drug release was 27% and 34% respectively from CS‐MMT‐NCQDs and CS‐MMT nanocarriers within 24 h at pH 7.4. Compared to CS‐MMT‐DOX, strong bonding between components and DOX in CS‐MMT‐NCQDs‐DOX decreased DOX entrapment at pH 7.4. Indeed, protonation of amine groups, swelling and degradation of hydrogel chains, and destabilization of nanocarrier structure resulted in more drug release for CS‐MMT‐DOX than CS‐MMT‐NCQDs‐DOX at pH 7.4. Moreover, a comparison of drug loading and entrapment efficiency with release results shows that the incorporation of NCQDs in the nanocarrier increases the drug loading, while drug retention in normal tissues is not compromised. This finding confirms the usefulness of CS‐MMT‐NCQDs‐DOX nanocarrier as a sustained release drug delivery system.

The faster drug release rate in the acidic environment for CS‐MMT‐NCQDs‐DOX nanocarriers is due to surface amino groups in NCQDs. In more detail, DOX and CS amino groups are protonated at pH 5.4. NCQDs with positively charged amine groups can increase the repulsive force between components and in turn lead to the deformation of CS‐MMT‐NCQDs hydrogel nanocarrier and the consequent increase in DOX release at pH 5.4. The protonated amino groups of CS and NCQDs in the lower pH (5.4) disrupted the electrostatic interactions between the nanocarrier components, resulting in an improved buffer penetration inside the nanocarrier matrix and consequently an enhanced release rate. The drug was released at a slower rate at pH 7.4 compared to pH 5.4, indicating an effective stimulus‐responsive performance of nanocarriers. Besides, the pH responsivity of the nanocarriers proves more drug release in the tumor microenvironment and less side effect risk of the fabricated drug delivery system [35, 71–73].

The article "Preparation of a pH‐responsive chitosan‐montmorillonite‐nitrogen‐doped carbon quantum dots nanocarrier for attenuating doxorubicin limitations in cancer therapy" was retracted in 2025. Reasons: duplicated images; duplicated data; unreliable results or conclusions; concerns about the data.

### 3.4 Kinetic modeling of drug release

Using data obtained from the dialysis method, we were able to evaluate the drug release kinetics. We used the correlation coefficient (*R* ^2^) to compare the models. The generated kinetic parameters are presented in Table 3. The release data at pH 5.4 fit Baker and First‐order models with higher *R* ^2^ values, whereas the drug release at pH 7.4 can be properly approximated by Hixon‐Crowellbio and Higuchi models. The value of *n* in the Korsmeyer‐Peppas model was implemented to investigate the drug release mechanism. Regarding spherical matrices, the *n*‐values below 0.43 suggest Fickian diffusion, while the *n* values above 0.85 indicate case‐II transport [74]. As can be seen in Table 3, while the *n*‐value is 0.8598 for the CS‐MMT‐NCQDs‐DOX nanocarrier at pH 7.4, this value is quantified about 0.3734 at pH 5.4. These results indicate that the drug release follows a controlled pattern at pH 5.4 [48]. The greatest values of rate constant for two pH values of 5.4 and 7.4 were 0.1910 (calculated according to Korsmeyer‐Peppas model) and 0.0816 (calculated according to Higuchi model), respectively, while the least values of the models' rate constant for pH of 5.4 and 7.4 were 0.0035 (calculated according to Baker model) and 0.0023 (calculated according to Baker model), respectively. Such large difference between greatest and least rate constants may also reinforced the possibility of DOX sustained release from the fabricated nanocarrier.

**TABLE 3:** The parameters and correlation coefficients of the kinetic models for estimating the release of DOX from CS‐MMT‐NCQDs nanocarrier at pH 5.4 and pH 7.4

		**First‐order**	**Higuchi**	**Hixson‐Crowell**	**Baker**	**Korsmeyer‐Peppas**
pH 5.4	*R* ^2^	0.9967	0.9637	0.9829	0.9955	0.9333
		*K*_1_ = 0.0255	*K_P_* = 0.1056	*K*_β_ = 0.0050	*K_C_* = 0.0035	*K_H_* = 0.1910 *n* = 0.3734
pH 7.4	*R* ^2^	0.9559	0.9966	0.9876	0.9341	0.9394
		*K*_1_ = 0.0246	*K_P_*_ _= 0.0816	*K*_β_ = 0.0056	*K_C_* = 0.0023	*K_H_* = 0.0243 *n* = 0.8598

### 3.5 In vitro cytotoxicity assay

The cytotoxicity effect of CS‐MMT‐NCQDs, CS‐MMT‐NCQDs‐DOX, and free drug on MCF‐7 cells was determined after incubation for 72 h employing the MTT assay shown in Figure 6. We used MCF‐7 cells that received no treatment as control. The drug concentration was 4.8 µg mL^−1^ in CS‐MMT‐NCQDs‐DOX and free DOX. Based on ISO standards, cell viability larger than 80% is acceptable for a biocompatible nanocarrier. The results showed that CS‐MMT‐NCQDs nanocarriers were biocompatible because the resultant viability percentage was more than 80% in MCF‐7 cells. Moreover, CS‐MMT did not induce significant cell death, which is consistent with Banik et al. report [75]. They used GA to chemically cross‐link carboxymethyl chitosan and montmorillonite and studied cell viability of carboxymethyl chitosan‐montmorillonite nanoparticles with varying concentrations of MMT and GA. They found that the nanoparticles did not significantly reduce viability percentage. All these findings lead us to conclude the nontoxicity of CS‐MMT hydrogel without NCQDs. As shown in Figure 6, the viability of treated cells with CS‐MMT‐NCQDs is less than that of treated cells with CS‐MMT, confirming the toxic effect of NCQDs on MCF‐7 cells. The induced cytotoxicity by the presence of NCQDs in CS‐MMT‐NCQDs hydrogel is in agreement with the results presented by Cutrim et al. [36]. They concluded that the 5‐Fluorouracil‐carbon quantum dots nanoconjugate system caused a higher decline in MCF‐7 viability as compared to free 5‐Fluorouracil. The cytotoxicity effect of CS‐MMT‐NCQDs‐DOX nanocarriers was more than that of free DOX and CS‐MMT‐DOX with *p* < 0.001. In more detail, the cell viability of free DOX, CS‐MMT‐DOX, and CS‐MMT‐NCQDs‐DOX was calculated at about 37%, 62%, and 24%, respectively. These findings offer compelling evidence on better uptake of fabricated CS‐MMT‐NCQDs nanocarrier due to the effective role of NCQDs for the improvement of DOX release. This result shows that drug‐loaded CS‐MMT‐NCQDs in comparison with free DOX released the drug over more prolonged time intervals for apoptotic induction, leading to more reduction in cell viability.

**FIGURE 6:** The viability analysis of MCF‐7 cells treated with CS‐MMT‐NCQDs, CS‐MMT‐NCQDs‐DOX, and free DOX groups after 72 h. Data are represented as mean ± SEM of three independent experiments in duplicate (** signifies *p*‐value ≤0.01 compared to control. *** signifies *p*‐value ≤0.001 compared to control. $$$ indicates *p*‐value ≤0.001 compared to free DOX)

The article "Preparation of a pH‐responsive chitosan‐montmorillonite‐nitrogen‐doped carbon quantum dots nanocarrier for attenuating doxorubicin limitations in cancer therapy" was retracted in 2025. Reasons: duplicated images; duplicated data; unreliable results or conclusions; concerns about the data.

### 3.6 Cell apoptosis study

We opted for the flow cytometry assay to determine the apoptotic and necrotic induction effect of CS‐MMT‐NCQDs, CS‐MMT‐DOX, CS‐MMT‐NCQDs‐DOX, and free DOX on MCF‐7 cells (Figure 7). The apoptotic rate was identified using Annexin V‐PI dual staining. In each density plot, there are four quadrants representing necrotic cells (V−/PI+; Q1), late apoptotic cells (V+/PI+; Q2), early apoptotic cells (V+/ PI−; Q3), and viable cells (V−/PI−; Q4). The cells treated with CS‐MMT‐NCQDs nanocarriers compared to the control group demonstrated less reduction in the percentage of viable cells (97.5%), proving the non‐toxicity and biocompatibility of the fabricated nanocarriers. This finding is in line with the MTT results discussed earlier. The cells treated with CS‐MMT‐NCQDs‐DOX showed a drastic rise in the percentage of necrotic cells as compared to CS‐MMT‐DOX and free DOX. This result highlights the better uptake achieved due to the presence of NCQDs [67]. The same result was observed in the study of the effect of poly (L‐histidine) based pH‐responsive micelles for intracellular DOX delivery against MCF‐7/ADR cells. DOX loaded poly (L‐histidine) based micelles enhanced cytotoxicity compared to free DOX [76]. The percentage of viable cells was lower in DOX than CS‐MMT‐DOX, but higher in DOX than CS‐MMT‐NCQDs‐DOX. All these findings are also in accord with the results discussed in the cytotoxicity study section.

**FIGURE 7:** Cytometry analyses of MCF‐7 cells treated with control (A), free DOX (B), CS‐MMT‐NCQDs (C), CS‐MMT‐DOX (D), and CS‐MMT‐NCQDs‐DOX (E). In cases where non‐gated cells in FL1 (Annexin V) versus FL3 (P.I.) channels were used, the fluorescence intensity of 5000 events was measured. The lower left quadrant cells are defined as viable, the lower right quadrant cells as apoptotic, the upper left as necrotic, and the upper right quadrant cells as late apoptotic.

To further make a comparison between flow cytometry results, we calculated cell inhibition in each sample as the summation of late and early apoptotic cell percentages. The inhibition percentages of treated cells with free DOX, CS‐MMT‐NCQDs, CS‐MMT‐DOX, and drug‐loaded CS‐MMT‐NCQDs nanocarriers respectively were 70.82%, 1.35%, 38.70%, and 90.30%. In comparison with DOX (13.5%), a smaller percentage of necrotic cells (1.06%) was achieved after the treatment of cells with CS‐MMT‐NCQDs‐DOX. As expected, these results revealed that drug‐loaded CS‐MMT‐NCQDs nanocarriers caused a meaningful inhibitory effect on the proliferation of MCF‐7 cells. Besides, the percentage of necrotic cells was small in CS‐MMT‐NCQDs‐DOX in comparison to free DOX. These findings support the enhanced sustained release of DOX from CS‐MMT‐NCQDs nanocarriers. These findings are consistent with the results concluded about the improved sustained release of drug loaded CS‐MMT‐NCQDs. In research done by Lee and co‐workers, the cell viability of 20%–30% resulted from the effect of pH‐responsive micelles, of which surface was decorated with folate containing DOX on MCF‐7 cells [9].

The article "Preparation of a pH‐responsive chitosan‐montmorillonite‐nitrogen‐doped carbon quantum dots nanocarrier for attenuating doxorubicin limitations in cancer therapy" was retracted in 2025. Reasons: duplicated images; duplicated data; unreliable results or conclusions; concerns about the data.

## 4 CONCLUDING REMARKS

In this paper, the DOX‐loaded CS‐MMT‐NCQDs hydrogel nanocomposite was loaded into water in oil in water double emulsions to attain improved loading, enhanced sustained release, and increased apoptosis induction. The application of CS‐MMT‐NCQDs hydrogel nanocomposite for loading DOX noticeably improved loading and entrapment efficiencies compared to previous research, highlighted the crucial role of NCQDs in the interaction with components. The results of FESEM, FTIR, and XRD verified the incorporation of all components into the fabricated nanocomposite. Furthermore, the controlled release of DOX was achieved from the application of double emulsions to develop DOX‐loaded CS‐MMT‐NCQDs nanocomposite. The release behavior of the fabricated platform is also pH‐responsive, which results from the interactions between the drug and nanocomposite components. Moreover, the evidence from cytotoxicity and apoptosis studies highlighted higher cytotoxicity and better uptake of CS‐MMT‐NCQDs‐DOX due to the effective role of NCQDs. According to the aforementioned results, this DOX delivery system can be a promising candidate for addressing DOX attributed defects such as low loading efficiency, poor sustained release, and adverse side effects on normal cells. Consequently, it is hoped that our research will be helpful in solving difficulties associated with DOX as an antitumor drug for cancer treatment.

## AUTHORS CONTRIBUTION

Erfan Rahmani: Investigation, methodology, and writing – original draft. Mehrab Pourmadadi: Formal analysis and funding acquisition. Sohrab Ali Ghorbanian: Formal analysis, investigation, and project administration. Fatemeh Yazdian: Project administration, supervision, and validation. Hamid Rashedi: Conceptualization, data curation, and supervision. Mona Navaei Nigjeh: Methodology, formal analysis, and resources.

## CONFLICT OF INTEREST

The authors have declared no conflict of interest.
